The article "SPOP Inhibition of Endometrial Carcinoma and Its Clinicopathological Relationship" was retracted in 2023. Reasons: signs of a paper mill; suspected computer-generated content; unreliable results or conclusions; concerns about the data.

# SPOP Inhibition of Endometrial Carcinoma and Its Clinicopathological Relationship

**DOI:** 10.1155/2022/5721630

**Published:** 2022-04-15

**Authors:** Qing Zhu, Guanghui Zhang, Mingyang Tang, Rumin Zheng, Huaiyong Gan

**Affiliations:** ^1^Department of Pathology, The First Affiliated Hospital of Bengbu Medical College, Bengbu, 233399 Anhui, China; ^2^Department of Pathology, Bengbu Medical College, Bengbu, 233030 Anhui, China; ^3^Class 2020, Clinical Pathology, The Graduate School, Bengbu Medical College, Bengbu, 233030 Anhui, China; ^4^Anhui Key Laboratory of Infection and Immunity, Bengbu Medical College, Bengbu, 233030 Anhui, China; ^5^Class 2019, Medical Imaging Technology, The Medical Imaging School, Bengbu Medical College, Bengbu, 233030 Anhui, China

## Abstract

**Objective:**

Endometrial carcinoma (EC) ranks first in the incidence of female genital malignancies in developed countries. SPOP (speckle-type POZ protein) has changed in EC with a statistically high frequency. This research may play a crucial role in the initiation and progression of EC, ultimately leading to fresh therapeutic targets. Explore the expression of SPOP in EC; observe its effect on the proliferation, invasion, and migration of EC cells after upregulating the expression of SPOP through RNA activation.

**Methods:**

The expression levels of SPOP protein in 150 EC tissues and 45 normal endometrial tissues were detected by immunohistochemistry and Western blotting. Analyze the relationship between SPOP expression and clinicopathological characteristics. The differences of the proliferation, migration, and invasion abilities between before and after transfection were analyzed using CCK-8 and Transwell assays.

**Results:**

The results of immunohistochemistry and Western blotting showed the expression level of SPOP in EC tissue significantly reduced or even missed compared with normal endometrial tissue. The results of CCK-8 showed that the growth of EC significantly slowed down after the upregulating of SPOP expression. The results of the Transwell assay showed the migration and invasion abilities of EC cells were weakened after the level of SPOP was upregulated.

**Conclusions:**

The expression level of SPOP in EC tissues is lower and related to the clinicopathological features compared with normal endometrial tissues. After upregulating the SPOP expression by RNA activation in EC cell lines, the abilities of proliferation, migration, and invasion of cells were significantly inhibited.

## 1. Introduction

Endometrial carcinoma is a malignant tumor derived from endometrial epithelial cells. It is more common in menopausal and postmenopausal women, and the incidence peaks at 55-65 years old. In recent years, due to the increase in the average life expectancy of the population and the application of hormone replacement therapy for menopause, the incidence rate is on the rise [1]. According to international treatment guidelines, patients with early-stage endometrial carcinoma can be cured with surgery or brachytherapy and/or external beam therapy alone, whereas patients with recurrent and locally or distantly metastasized endometrial carcinoma are limited by disease progression and treatment modalities. The prognosis is poor, and the 5-year survival rate of patients with distant metastasis is less than 20% [2]. Although surgery, radiotherapy, and chemotherapy can obtain certain survival benefits for patients, their drug resistance, metastasis, and recurrence still seriously threaten the life and health of patients. Therefore, in-depth understanding of the occurrence and development mechanism of endometrial carcinoma and the study of endometrial carcinoma-related target genes provide a theoretical basis for the diagnosis and treatment of endometrial carcinoma [3]. Studies have found that E3 ubiquitin ligase speckle-type POZ protein (SPOP) plays an important inhibitory role in the occurrence and development of EC [4]. SPOP belongs to a class of protein called ubiquitin ligase, which exists in human tissues and is highly conserved. SPOP is a new type of tumor suppressor gene, which is located at 17q21 in the human chromosome [5]. It has a high deletion rate and loss of heterozygosity in tumor cells, and it has the function of significantly inhibiting tumor growth and spread [6]. A number of SPOP-related research results suggest that SPOP has antitumor function and is an important cancer gene in 21 different types of cancer. SPOP target proteins are involved in a variety of important cellular functions, and SPOP is involved in cancer formation by mediating the stability of target proteins. It has also been reported that SPOP acts as a ubiquitin ligase to inhibit tumor by ubiquitinating and degrading the level of malignant tumor protein SRC-3/AIB1 [7]. RNA activation (RNAa) introduces double-stranded RNA molecules (dsRNA) to the promoter region of the gene into tumor cells. RNAa is an Argonaute protein guided by small double-stranded RNA to involved transcriptional gene activation mechanism, and strand RNA is called small activating RNA (saRNA) [8]. This study detects the expression of the SPOP gene in EC and its correlation with clinicopathological factors and intends to use RNA activation to upregulate the expression of the SPOP gene in human EC cell lines (Ishikawa, ISK) and explore its effect on the proliferation, invasion, and migration of EC cells. It may provide a new idea for the occurrence, development, diagnosis, treatment, and prognosis of endometrial carcinoma.

## 2. Material and Methods

### 2.1. Patient and Control Selection

The experimental group was EC tissue, which was confirmed as type I EC (i.e., endometrioid carcinoma) by routine pathological examination after the operation. We selected 150 patients who were 27 to 81 years old from January 2018 to December 2019. According to the 2019 FIGO standard, in the clinicopathological staging, 89 patients were from stage I to II and 61 patients were from stage III to IV. According to the 2014 WHO standard, the histological grades were G1 for 42 patients, G2 for 72 patients, and G3 for 36 patients. There were 79 patients with muscular layer infiltration ≤ 1/2 and 71 patients >1/2. There were 54 patients with lymph node metastasis and 96 patients without lymph node metastasis. They did not receive anticarcinoma treatment before surgery and had complete clinical data. The mean age was 54.52 ± 5.79 years. The pathological diagnosis was reviewed by two pathology experts. The standards refer to the latest classification standards of the International Association of Gynecological Pathologists and the World Health Organization [9]. The control group was normal endometrial (NE) tissue; we selected 45 patients who perform a gynecological biopsy of the endometrial tissue or hysterectomy due to other benign diseases. All tissues came from the Pathology Department, the First Affiliated Hospital of Bengbu Medical College.

### 2.2. Immunohistochemical Staining

Automatic microtome slices the wax block into 0.5 *μ*m thick slices. After dewaxing, perform antigen retrieval in 121°C citrate solution for 3 minutes. After natural cooling, let it stand in 3% H_2_O_2_ solution for 10 minutes; the anti-SPOP rabbit anti-human primary antibody was washed at 60°C for 1 h, washed with PBS for 3 × 6 min; the secondary antibody was flown at 37°C for 30 min. After washing with PBS, DAB developed color. Observe under the microscope. The SPOP protein is mainly located in the cytoplasm and nucleus. The yellow particles in the cytoplasm or nucleus of the antibody are used as a positive signal to comprehensively score the intensity of cell staining and the percentage of positive cells. The following are the scores according to staining intensity: colorless is 0 point, light yellow is 1 point, brownish yellow is 2 point, and brown is 3 point, and they are scored based on the percentage of positive cells: 0 point means no positive cells, positive cells ≤ 10% is 1 point, 11% to 50% for positive cells is 2 points, 51% to 75% for positive cells is 3 points, and positive cells > 75% is 4 points; the product of staining intensity and percentage of positive cells ≥ 2 is considered positive for immunoreaction and that of positive cells < 2 is divided into decreased expression or negative immune response [10]. Image analysis was performed using Image-Pro Plus software, and the expression of SPOP protein was judged by integrating optical density (IOD)/area values.

### 2.3. Cell Lines and Main Reagents

Human EC cell line ISK, construction of SPOP-saRNA expression vector, reverse transcription kit, and PCR kit are from Shanghai Jima; DMEM (high) culture medium, PBS balance solution, and fetal bovine serum from Hyclone; SPOP antibody from Abcam, ab137537; anti-GAPDH antibody from Abcam, ab8245; LipofectamineTM2000 and Trizol reagent from Invitrogen; CCK-8 reagent and Transwell chamber from Biyuntian; and Binding Matrigel from Matrigel, BD.

### 2.4. Cell Culture

The ISK cells were cultured in a 37°C, 5% CO_2_ incubator; the cells grew adherently and were passaged every 2 to 3 days. The old culture medium was discarded during the passage, washed with PBS 2 to 3 times, and added trypsinization digestion. Add culture fluid and pipette the cells; reset the cell fluid to inoculate the culture bottle. The experiment takes cells in the logarithmic growth phase.

### 2.5. Sequence Design and Synthesis of saRNA

Against oligonucleotide synthesized at the target site, according to the role of transcription RNA and RNA activation (saRNA) design principles, design, and synthesis, select one target: 796-1869, AACATCTGCCTAGATCGGCTA; GC content is 51.67%. Against oligonucleotide synthesized at the target site. The saRNA sequences are as follows: dsSPOP—5′-GCT TAA GCG GGA ACG AAT AAT-3′; 5′-TTA ACC GGT AAT CGG CGC CGC-3′; control—5′-CCG GAA TTC CGG ATT ACG ACG-3′; 5′-AATTGG CCC TAA TCG GCC GTA-3′.

### 2.6. Cell Transfection and Grouping

Before transfection, inoculate a 6-well plate at 2 × 10^5^ cells/well, and start transfection when the cell density reaches 70% to 80%. The transfection steps are carried out according to the instructions of the Lipofectamine™ 2000 reagent. The final concentration of dsSPOP is 50 nmol/L. After 48 hours of incubation, dsSPOP was transfected into ISK cells. The following are the groups: experimental group (transfected with dsSPOP), negative control (NC) group (transfected with disordered RNA), and blank control (BC) group (not transfected).

### 2.7. Western Blotting

In the cell transfection after 48 hours, each group of the cells was collected to extract proteins, and the proteins were separated with 10% polyacrylamide gel. Prepare separation gel and layering gel, and add the same amount of protein sample to each well for electrophoresis and sealing. Put the membrane in the diluted primary antibody (diluted 1 : 3000), shake gently for 2 h, then place in a 4°C refrigerator overnight, wash the membrane in TBST solution for 3 × 10 min, shake gently in the secondary antibody for 2 h, and wash the membrane in TBST solution for 3 × 10 min. Expose and develop the film after treatment with a developing solution; the gray value analysis is performed by the gel imaging system, and the experiment is repeated three times.

### 2.8. RT-PCR

In the cell transfection after 48 hours, each group of the cells of the total RNA was extracted with Trizol reagent and accurately quantified with an ultraviolet spectrophotometer. Take 5 *μ*g of total RNA for reverse transcription reaction. The following are the primer sequences: SPOP—upstream primer 5′-TCC TGA GCC TTC TCC ATC GTA-3′, downstream primer 5′-AGT GAC TTT CAT CTG GGC GTC-3′; GAPDH—upstream primer 5′-TTG TTG TAC TCT AAC GGT ACG-3′, downstream primer 5′-TCA CCC CAC CGA AAA TCC TAT-3′; PCR amplification reaction conditions are as follows: 95°C denaturation of 3 min; cycle 35 times according to the following parameters: 95°C denaturation of 40 s, 58°C anneal for 40 s, extend at 75°C for 40 s, and finally incubate at 75°C for 15 min. Take 5 *μ*L of PCR product, and perform gel electrophoresis for 30 min. Observe the DNA bands under ultraviolet light, take pictures, and analyze the gray value with the gel image processing system, and repeat the experiment three times.

### 2.9. CCK-8

Take the cells in the logarithmic growth phase, adjust the cell concentration to 4 × 10^5^ cells/mL, inoculate them in a 96-well plate, seed 150 *μ*L of cells fluid per well, incubate in a cell incubator for 24 h, and then transfect. Respectively, at 24, 48, 72, 96, and 120 h, add 20 *μ*L of CCK-8 reagents to each well and continue to incubate for 4 h. The microplate reader measures the optical density (OD) value of each well at 450 nm, and the experiment is repeated three times.

### 2.10. Cell Invasion and Migration Experiments

In the invasion experiment, 50 *μ*L of Matrigel per well was evenly spread on the membrane of the Transwell chamber. In the cell transfection after 48 hours, each group of the cells was digested into a cell suspension, the cell concentration was adjusted to 4 × 10^5^ cells/mL, and 200 *μ*L of the cells was taken. Take 200 *μ*L of cell suspension into the Transwell chamber, and place the chamber in the medium of a 24-well plate. After incubating for 24 hours, remove the Transwell chamber, wipe off the upper cells of the filter membrane with a cotton swab, fix the filter membrane with methanol, and add an appropriate amount of crystal violet solution for staining. Count the number of cells passing through the membrane in different random fields of view under the 400x eyepiece, and take the average value. Migration experiment Transwell chamber membrane is not covered with Matrigel. After the cells are transfected for 48 hours, the rest of the steps are the same as the invasion experiment. Each group has 3 chambers in parallel, and the experiment is repeated three times.

### 2.11. Statistical Analysis

The Statistical Package for Social Sciences (version 24.0) (SPSS Inc., Chicago, IL, USA) was used for statistical analysis. The two independent-sample *t*-test was used to compare the mean values of two independent continuous variables. The chi-square test was used to test the relationship between two categorical variables. SPOP and other individual group parameters were assessed using one-sample Kolmogorov–Smirnov *Z* test and found to be abnormally distributed. The statistical comparisons between groups were performed using the nonparametric Mann–Whitney *U* test. Data are presented as median (range). Statistical significance was defined as *P* < 0.05 for all comparisons.

## 3. Results

### 3.1. Immunohistochemical Staining

The results showed positive staining expressions in the cytoplasm of NE tissue, and the positive staining expression in the cytoplasm of EC tissue was weakened or even absent (*P* < 0.05) (Figure 1, Table 1).

### 3.2. The Relationship between SPOP Expression and Clinicopathological Factors of EC

According to the 2019 FIGO standard [9], in the clinicopathological staging, 89 patients were from stage I to II and 61 patients were from stage III to IV. According to the 2014 WHO standard, the histological grades were G1 for 42 patients, G2 for 72 patients, and G3 for 36 patients. There were 79 patients with muscular layer infiltration ≤ 1/2 and 71 patients > 1/2. There were 54 patients with lymph node metastasis and 96 patients without lymph node metastasis.

There was no significant correlation between the expression rate and age (*P* > 0.05). The positive rate of SPOP expression in EC FIGO stage III+IV was higher than that in FIGO stage I+II; muscular layer infiltration > 1/2 was higher than muscular layer infiltration ≤ 1/2; having lymph node metastasis was higher than not having lymph node metastasis (*P* < 0.05~*P* < 0.01) (Table 2).

### 3.3. Western Blotting Detection

Compared with that in EC, the expression of SPOP protein in NE is significantly higher (*P* < 0.01) (Figure 2). After 48 h cell transfection, compared with those in the NC group and the BC group, the expression of SPOP protein in the experimental group was significantly higher (*P* < 0.01) (Figure 2).

### 3.4. RT-PCR Detection

After 48 h cell transfection, the mRNA expression level of the experimental group was significantly higher than those of the NC group and the BC group (*P* < 0.01) (Figure 3).

### 3.5. The Effect of dsSPOP on the Activity of EC Cells

The CCK-8 test results showed that the cells were transfected for 24, 48, 72, 96, and 120 h; the inhibition rates were 5.3%, 15.6%, 37.2%, 43.3%, and 54.8%, respectively; compared with that of the NC group, the cell proliferation of the experimental group slowed down and the growth obviously suppressed (*P* < 0.05) (Figure 4).

### 3.6. The Effect of dsSPOP on the Invasion and Migration of EC Cells

The Transwell chamber experiment showed that compared with those of the BC group and the NC group, the cell invasion and migration ability of the experimental group were significantly reduced (*P* < 0.001) (Figure 5).

## 4. Discussion

In the current study, we found that SPOP expression in endometrial carcinoma tissues was remarkably decreased. In addition, SPOP activities by saRNA significantly inhibited endometrial carcinoma proliferation and metastasis, which may be related to the downregulation of MMP protein expression and inhibition of EMT.

EC has a high incidence and low cure rate in the world [1, 11]. Scientists have also been committed to the pathogenesis of this tumor, hoping to provide help for its diagnosis, treatment, and prognosis on the molecular level [12]. Tumor occurrence, development with abnormal activation of oncogenes, the inactivation of tumor suppressor genes, and DNA mismatch repair gene abnormalities are closely related [13, 14]. RNAa is one of the most popular technologies in the field of gene function and therapy in recent years. RNAa inhibits tumor growth by selectively activating or enhancing the expression of a specific tumor suppressor gene, without the need to find specific tumor-causing genes [15]. RNAa effects do not involve the degradation of any target sequence, through the recruitment of transcription activators, the activation of the gene transcription process, and the activation of chromatin modifications are caused [16]. Therefore, RNAa has almost unlimited target genes, increasing the total abundance of target gene mRNA, while retaining the diversity of natural splicing isoforms of mRNA [17]. It plays a role at the transcriptional and epigenetic level; therefore, it can activate the target gene permanently without changing the genome. The discovery could lead to a pioneering expansion of treatments for carcinoma and metabolic [18] and genetic diseases [19].

In this study, we applied immunohistochemistry and Western blotting on 150 cases of EC tissues and 45 cases of normal endometrial tissues. The results showed that the positive expression rate of SPOP protein in EC was 23.33%, compared with 82.22% in the endometrial tissue; the positive expression rate was significantly reduced. The expression of SPOP protein in two different endometrial tissues was statistically significant (*P* < 0.05), indicating that as the endometrial tissue progresses to carcinoma tissue, the positive expression rate of SPOP was significantly reduced, and the SPOP protein was obviously related to the occurrence and development of EC. The expression of SPOP in EC was significantly correlated with tumor histological grade, clinical stage, muscular layer infiltration, and lymph node metastasis (*P* < 0.05 to *P* < 0.01).

CCK-8 kit detects cell proliferation in human EC cells after SPOP gene RNA is activated. The results show that the cell growth of the experimental group is significantly slower than that of the negative group, indicating that the SPOP gene is activated for EC cell doubling time was significantly prolonged. Transwell chamber experiment is a better way to study tumor cell invasion and migration. It can simulate the process of tumor cells digesting the matrix and traversing the barrier to invade and migrate. The experimental results show that after SPOP expression is activated, the EC cells that can cross the barrier are significantly reduced compared with the NC group and BC group. This indicates that the invasion and migration ability of EC cells is inhibited, confirming that the SPOP gene is associated with human endometrial cells. The proliferation of carcinoma cells is closely related to invasion and metastasis. In a normal human body, proteins that regulate cell proliferation and viability need to be expressed in a timely manner and accurately modified to maintain their normal functions. When these proteins are abnormally expressed or modified, they may lead to excessive cell proliferation and cause cell canceration. Therefore, in order to prevent this phenomenon, these proteins need to be effectively degraded through a certain pathway [20]. Studies have shown that the degradation of intracellular target proteins is mainly completed by the ubiquitin-proteasome system (UPS), a UPS that exists in a multicatalytic cytoplasmic and nuclear protein complex in all eukaryotic cells, mainly responsible for the proteolysis of nonlysosomal pathways and maintaining normal protein homeostasis in cells. It is composed of ubiquitin (Ub), ubiquitin-activating enzymes (E1), ubiquitin-conjugating enzyme (E2), ubiquitin-protein ligase (E3), 26S proteasome, and deubiquitinating enzymes (DUBs). SPOP is an adaptor protein of Cullin3 (Cul3) family E3 ubiquitin ligase, and many studies have demonstrated the association between its mutation and endometrial carcinogenesis [21].

SPOP protein is the adaptor protein of Cullin3 family E3 ubiquitin ligase; it is a member of the MATH-BTB nuclear protein family [22, 23]. The SPOP gene is located on the human chromosome 17q21.33. The SPOP protein consists of 374 amino acid residues and has a relative molecular mass of 42,000 [5]. The encoded SPOP protein is an essential substance that mediates protein ubiquitination. Ubiquitination is one of the main ways of protein degradation, which is maintaining the normal physiological functions of cells [24]. The abnormal regulation of the ubiquitination system plays an essential role in the occurrence and evolution of tumors. Many studies have shown that SPOP protein is a vital factor in studying tumor mechanisms, and its role in the event and development of tumors is more complex [25, 26]. A study found that SPOP protein can degrade the expression level of malignant tumor protein SRC-3/AIB1 through ubiquitination, thereby inhibiting the growth and spread of tumors and exerting a tumor suppressor effect [27]. As a linking molecule of E3 ubiquitin ligase Cullin 3-RING box, SPOP mainly binds to CUL-3 through the BTB/POZ domain to form a SPOP/CUL complex, which connects ubiquitin to a specific site of the target protein. Substrate proteins containing the SBC domain are ubiquitinated and degraded, such as steroid receptor coactivator-3 (SRC-3) [28]. However, studies have also shown that SPOP protein degrades breast carcinoma metastasis inhibitor (BRMS1) through ubiquitination, promoting tumor cell metastasis [29]. Breast cancer metastasis suppressor 1 (BRMS1) is an important factor in inhibiting breast cancer metastasis. Cullin 3 (Cul3), a component of E3 ubiquitin ligase, enhances the metastatic ability of breast cancer by promoting the degradation of BRMS1 protein. The interaction is mediated by the SPOP adaptor protein [30]. This study indicates the SPOP protein is lowly expressed in EC tissues. In contrast, it is highly expressed in normal endometrial tissues, suggesting that SPOP protein may participate in EC by mediating the protein ubiquitination of EC cells [31]. It can be seen that with the continuous advancement of research, an in-depth study of the expression and signal pathways of SPOP-related oncogenes and tumor suppressor gene products in EC tissues will be more helpful to understand the regulatory role of SPOP in the occurrence and evolution of EC [32].

In this study, we applied immunohistochemistry and Western blotting on 150 cases of EC tissues and 45 cases of normal endometrial tissues. The results showed that the positive expression rate of SPOP protein in EC was 23.33%, compared with 82.22% in the endometrial tissue; the positive expression rate was significantly reduced. The expression of SPOP protein in two different endometrial tissues was statistically significant (*P* < 0.05), indicating that as the endometrial tissue progresses to carcinoma tissue, the positive expression rate of SPOP was significantly reduced, and the SPOP protein was obviously related to the occurrence and development of EC. The expression of SPOP in EC was significantly correlated with tumor histological grade, clinical stage, muscular layer infiltration, and lymph node metastasis (*P* < 0.05 to *P* < 0.01).CCK-8 kit detects cell proliferation in human EC cells after SPOP gene RNA is activated. The results show that the cell growth of the experimental group is significantly slower than that of the negative group, indicating that the SPOP gene is activated for EC cell doubling time was significantly prolonged. Transwell chamber experiment is a better way to study tumor cell invasion and migration. It can simulate the process of tumor cells digesting the matrix and traversing the barrier to invade and migrate. The experimental results show that after SPOP expression is activated, the EC cells that can cross the barrier are significantly reduced compared with the NC group and BC group. This indicates that the invasion and migration ability of EC cells is inhibited, confirming that the SPOP gene is associated with human endometrial cells. The proliferation of carcinoma cells is closely related to invasion and metastasis.

## 5. Conclusions

This study showed that the loss of SPOP gene expression is closely related to the occurrence and development of EC. The detection of its expression level has a specific reference value for the early diagnosis, clinical progress and prognosis of EC [33, 34]. Through multifactor analysis, explore the inhibitory effect of SPOP gene in human EC and the risk factors of EC metastasis, and provide more accurate means for disease monitoring and screening of high-risk groups [35]. Its detection will help to improve the accuracy and objectivity of diagnosis; it has particular guiding significance for the prognostic evaluation, follow-up, and appropriate treatment of EC.

## Figures and Tables

**Figure 1:** The expression of SPOP in different endometrial tissues (scale bar, 20 *μ*m). (a) SPOP is positively expressed in the cytoplasm of endometrial tissue (×100). (b) Negative expression of SPOP in EC (×100).

**Figure 2:** SPOP-saRNA reduced Ishikawa cell proliferation. (Western blotting detects the expression of the SPOP gene in different endometrial tissues. Representative images for SPOP are shown.)

**Figure 3:** RT-PCR detects SPOP gene protein expression.

**Figure 4:** CCK-8 detects ISK proliferation.

**Figure 5:** The influence of SPOP on the invasion and migration ability of ISK cells.

**Table 1:** Expression of SPOP in distinct tissue types.

Histological type	SPOP			
	Cases	Negative	Positive	*P*
NC tissues	45	8	37	
EC tissues	150	115	35	<0.01

**Table 2:** The association of SPOP expression with clinicopathological features in EC.

	SPOP			
Factor	Cases	Negative	Positive	*P*
Age				
<50	42	29	13	
≥50	108	86	22	0.169
Histological grade				
G1	42	18	24	
G2	72	66	6	
G3	36	31	5	<0.01
FIGO stage				
I+II	89	60	25	
III+IV	61	55	10	0.044
Muscular layer infiltration				
≤1/2	79	53	26	
>1/2	71	62	9	0.003
Lymph node metastasis				
No	96	69	28	
Yes	54	46	7	0.030

## Data Availability

The data used to support the findings of this study are available from the corresponding author upon request.
